# Efficient Reinforcement Learning from Demonstration via Bayesian Network-Based Knowledge Extraction

**DOI:** 10.1155/2021/7588221

**Published:** 2021-09-24

**Authors:** Yichuan Zhang, Yixing Lan, Qiang Fang, Xin Xu, Junxiang Li, Yujun Zeng

**Affiliations:** College of Intelligence Science and Technology, National University of Defense Technology, Changsha, China

## Abstract

Reinforcement learning from demonstration (RLfD) is considered to be a promising approach to improve reinforcement learning (RL) by leveraging expert demonstrations as the additional decision-making guidance. However, most existing RLfD methods only regard demonstrations as low-level knowledge instances under a certain task. Demonstrations are generally used to either provide additional rewards or pretrain the neural network-based RL policy in a supervised manner, usually resulting in poor generalization capability and weak robustness performance. Considering that human knowledge is not only interpretable but also suitable for generalization, we propose to exploit the potential of demonstrations by extracting knowledge from them via Bayesian networks and develop a novel RLfD method called Reinforcement Learning from demonstration via Bayesian Network-based Knowledge (RLBNK). The proposed RLBNK method takes advantage of node influence with the Wasserstein distance metric (NIW) algorithm to obtain abstract concepts from demonstrations and then a Bayesian network conducts knowledge learning and inference based on the abstract data set, which will yield the coarse policy with corresponding confidence. Once the coarse policy's confidence is low, another RL-based refine module will further optimize and fine-tune the policy to form a (near) optimal hybrid policy. Experimental results show that the proposed RLBNK method improves the learning efficiency of corresponding baseline RL algorithms under both normal and sparse reward settings. Furthermore, we demonstrate that our RLBNK method delivers better generalization capability and robustness than baseline methods.

## 1. Introduction

Recent research on reinforcement learning (RL) has made impressive achievements in various domains, including video gaming [1], stock trading [2], and recommendation systems [3]. However, the resource-exhausting training seriously hinders the deployment of RL in real-world scenarios. One of the most important reasons for this issue is that RL agents have no background knowledge and have to learn from scratch, which is neither efficient nor realistic. In contrast, during the human learning process, we expect to learn new tasks by watching demonstrations first, and this inspires the research on reinforcement learning from demonstration (RLfD) [4], which has been proved to be promising in robot grasping [5] and unmanned vehicle driving [6], etc.

However, most previous RLfD methods do not take full advantage of expert demonstrations, limited by treating them as the accurate behavioral templates without providing insight into the reasons of performing such actions. Demonstrations in these RLfD methods are regarded as the low-level representation of human knowledge, which restrains their generalization capability [7]. Moreover, neural network-based RLfD methods aforementioned have limited interpretability, and they also lack the ability of acting robustly to the observation disturbance.

Considering that obtaining expert demonstrations is costly, it is essential to explore how these demonstrations can be used effectively. Therefore, a superior RLfD method should be able to extract knowledge from demonstrations that not only improves the algorithm performance for the same task but also provides explanations of the demonstrator's actions, which facilitates the generalization of the final learned behavioral policy. Here, following the definition proposed in [8], we treat “knowledge” as validated information about the relationships between entities in a certain context and the theoretical definition will be introduced in Section 4.2. Although such knowledge is generally efficient and concise, it is usually uncertain, coarse, and difficult to be expressed or quantified, which indicates that it needs to be further fine-tuned and adjusted to fully accomplish the target task.

As a probabilistic graphical model, Bayesian networks [9] can be used as an appropriate pattern to exploit task-agnostic knowledge from demonstrations since they have multiple advantages. Firstly, as a kind of probabilistic model, Bayesian networks can learn and represent uncertain and coarse knowledge to accomplish probabilistic reasoning. Besides, Bayesian networks have directed graph structures in which the nodes represent real-world observations and actions and the weights between nodes are conditional probability values used to quantify causal relationships between nodes. Thus, Bayesian networks are easy to be interpreted, which provides transparent insight into the extracted knowledge. Moreover, Bayesian networks can provide confidence in decision-making process compared to commonly used methods.

Inspired by the aforementioned ideas, we propose a novel RLfD method called Reinforcement Learning from demonstration via Bayesian Network-based Knowledge (RLBNK) that extracts probabilistic knowledge from expert demonstrations via Bayesian networks and combines the knowledge with RL. The RLBNK method aims to learn a hybrid policy that consists of a fixed knowledge module represented by a Bayesian network and a trainable refine module represented by a neural network, where the refine module undertakes the role of refining the probabilistic coarse knowledge represented by the Bayesian network. By leveraging Bayesian networks as the knowledge representation pattern, the agent can quantify the uncertainty of the prior knowledge extracted from demonstrations, which guides the employment of the probabilistic knowledge. More specifically, we propose two variant RLBNK methods called RLBNK-concat and RLBNK-switch. For RLBNK-concat, the agent concatenates the decision confidence vector provided by the Bayesian network to the current state vector as input and optimizes the whole policy by RL. In this method, the decision confidence vector implicitly provides instruction to the agent. As for RLBNK-switch, it divides the state space according to the decision confidence vector provided by the pretrained Bayesian network knowledge module: if the decision confidence is high, the decision will be made by the Bayesian network; otherwise, the decision will be made by the neural network-based refinement module. Note that for both variants, the knowledge module represented by the Bayesian network is fixed during the RL process. Simulation results illustrate that our RLBNK outperforms the well-established baselines in terms of data efficiency, generalization capability, and robustness.

In summary, the main contributions of this paper are threefold:

1. An influence-based state abstraction algorithm NIW is proposed to obtain conceptional abstract states from original expert demonstrations. And Bayesian networks then extract probabilistic coarse knowledge from these abstract demonstrations.
2. A novel RLfD method called RLBNK is proposed, which composes of a Bayesian network that represents probabilistic coarse knowledge and a neural network-based refine module that refines the prior knowledge. And the advantages of RLBNK are also analysed and discussed.
3. Extensive experiments are conducted to verify the effectiveness of the RLBNK method. The results show that the RLBNK method can achieve better performance in data efficiency, generalization capability, and robustness than the baseline methods.

The remainder of this paper is structured as follows.  Section 2 and Section 3 introduce the related works and preliminaries of this paper. The methodology of the RLBNK and the corresponding analysis and discussion are presented in Section 4. Finally, the experimental results are illustrated and analysed in Section 5.  Section 6 concludes this paper and envisions the future work.

## 2. Related Work

### 2.1. Reinforcement Learning from Demonstration

Reinforcement learning from demonstration (RLfD) is considered as an important branch of learning from demonstration (LfD) method that combines demonstrations with conventional RL to improve the sample efficiency [10] in the training process. Existing RLfD methods are basically rooted in the following three ideas: (1) policy pretraining; (2) reward shaping; (3) providing auxiliary loss.

Policy pretraining [6] is the most commonly used RLfD method in practice. It pretrains the RL policy with demonstrations in a supervised manner via behavior cloning [11], then proceeding with regular RL. The typical work following this idea is the AlphaGo algorithm [12]. However, this approach cannot guarantee the exploration quality during the proceeding policy optimization process, which usually results in “catastrophic forgetting” [13]. Moreover, neural networks are often apt to overfit the demonstrations, which impedes the generalization of the pretrained policy.

Reward shaping aims to instruct the agent's learning by constructing additional reward signals from expert demonstrations [14, 15]. With additional rewards, RL agents can learn more effectively by obtaining heuristic feedback from both the environment and the introduced rewards. For example, the soft Q imitation learning (SQIL) algorithm [15] stores demonstrations in the replay buffer and assigns a positive reward to them. The study [14] trains a supervised neural network from demonstration to act as a shaping function. However, this idea remains in the tendency of implicitly replicating the expert's action by encouraging the agent to explore the state space that is covered by the demonstrations.

Providing extra loss terms derived from demonstrations for RL policy function or value function optimization is the third mainstream idea of RLfD. For instance, deep Q-learning from demonstration (DQfD) [16] introduces demonstrations into deep Q-network (DQN) [1] by storing demonstration data into the experience replay buffer to pretrain the Q-network with different loss terms. Then, in the RL process, a prioritized sampling mechanism is employed to select experience data from the replay buffer for Q-network optimization. Likewise, the deep deterministic policy gradient from demonstration (DDPGfD) algorithm [5] inherits this idea and takes deep deterministic policy gradient (DDPG) [17] as the basic algorithm to extend DQfD to robot control tasks with continuous actions. Similar to the reward shaping idea, this approach also aims to encourage the agent to copy the expert's actions by constraining the objective of the optimization.

### 2.2. Imitation Learning

Imitation learning (IL) also utilizes demonstrations to acquire expert-like policies, and it can be broadly classified into behavioral cloning (BC) and inverse reinforcement learning (IRL). BC [11, 12, 18] is the most common imitation learning paradigm as the expert policy is extracted through supervised learning. However, the policies learned via BC suffer from the compounding error caused by covariate shift [19] in sequential decision-making tasks. Thus, the agent may easily drift away from the demonstrated states. The other IL paradigm is IRL, which tries to recover the reward function of the task by regarding the expert demonstrations are optimal and then learns policies within the RL framework. Thus, this IRL method can avoid compounding error occurs in BC. Combining the idea of generative adversarial networks (GANs) [20] and IRL, the generative adversarial imitation learning (GAIL) [21] method leverages adversarial training to learn the policy from demonstrations directly.

However, it is important to note that even though IL and RLfD are similar, there are fundamental differences between them. RLfD methods still assume access to the reward feedbacks from the environment even though they have the assistance from expert demonstrations, while IL methods do not rely on any reward signal [11, 18] or it constructs the reward function from demonstrations itself [21].

### 2.3. Knowledge Representation and Integration

Various typical patterns have been explored to represent prior knowledge, such as fuzzy methods [22, 23], rules [24–26], decision trees [27, 28], neural networks [11], and graphs [29, 30]. The advantage of fuzzy methods and rules is that they are naturally interpretable. However, it requires considerable human efforts to manually define the forms of rules and they are limited to represent complex relationships. In contrast, neural networks have powerful representation ability, but the lack of interpretability impedes their adoption. Graphs and decision trees are ideal tools for interpretable knowledge extraction and representation which can automatically extract knowledge from data. Compared to trees, Bayesian networks provide a more concise probabilistic representation as graph models, which are more in line with the human form of learning and reasoning.

There is also some research on the integration of knowledge into RL in different forms. The knowledge guided policy network (KoGuN) method [26] employs fuzzy rules as the knowledge controller. Fuzzy rules are difficult to extract knowledge from the data, and the membership function must be defined manually. Compared with fuzzy rules, Bayesian networks can extract the probabilistic knowledge with minimal human efforts. The requesting confidence-moderated policy advice (RCMP) algorithm [31] also utilizes uncertainty to guide the RL, where the uncertainty used in this algorithm is obtained by computing the variance of multiple Q-value vectors provided by a multiheaded Q-network. Then, the RCMP algorithm requires action advices from the online expert when it has high decision uncertainty. Therefore, this algorithm requires continuous instructions from an online expert.

## 3. Preliminary

### 3.1. Reinforcement Learning

RL aims to solve a sequential decision-making problem, where an RL agent optimizes its policy by interacting with the environment following a Markov decision process (MDP) [32]. A standard MDP ℳ is defined by a tuple 〈*𝒮*, *𝒜*, ℛ, *𝒫*, *γ*〉. Particularly, *𝒮* and *𝒜* are the state space and action space with sizes are |*𝒮*| and |*𝒜*|, respectively; ℛ represents the reward distribution function, with *r*_*t*_=*r*(*s*_*t*_, *a*_*t*_) is the immediate reward for taking action *a*_*t*_ in state *s*_*t*_ at timestep *t*; *𝒫* denotes the transition probability function, with Pr(*s*_*t*+1_*|s*_*t*_, *a*_*t*_) indicates the probability of transitioning from *s*_*t*_ to *s*_*t*+1_ upon action *a*_*t*_; *γ* ∈ (0,1] denotes the discount factor.

As shown in Figure 1, given a policy *π*, the RL agent chooses an action *a*_*t*_ according to *π*(*s*_*t*_) and then transits to the next state *s*_*t*+1_ following *Pr*(*s*_*t*+1_*|s*_*t*_, *a*_*t*_) and receives an instant reward *r*_*t*_. We define *R*_*t*_=∑_*k*=0_^*∞*^*γ*^*k*^*r*_*t*+*k*+1_ as the total discounted reward at *s*_*t*_ with discounted factor *γ*. The objective of an RL agent is to obtain the (near) optimal policy *π*^*∗*^ that maximizes the expectation of *R*_*t*_. Assuming that the policy network is parameterized by *ϕ*, the value function *V*^*π*_*ϕ*_^(*s*) is usually used to evaluate the policy *π*_*ϕ*_, where *V*^*π*_*ϕ*_^(*s*) can be defined as

(1) $$\begin{array}{c} V^{\pi_{\phi }}\left(s\right)=E^{\pi_{\phi }}\left[R_{t}|s_{t}=s\right], \end{array}$$

and the action value function *Q*^*π*_*ϕ*_^(*s*, *a*) is defined as

(2) $$\begin{array}{c} Q^{\pi_{\phi }}\left(s,a\right)=E^{\pi_{\phi }}\left[R_{t}|s_{t}=s,a_{t}=a\right], \end{array}$$

where *𝔼*^*π*_*ϕ*_^[·] denotes the expectation with respect to *π*_*ϕ*_.

The policy-based RL methods update the policy parameter *ϕ* via gradient ascent given by

(3) $$\begin{array}{c} \phi ⟵\phi +\alpha \nabla J\left(\phi \right), \end{array}$$

where *α* is the learning rate and *J*(*ϕ*) is the total expected reward that can be estimated by

(4) $$\begin{array}{c} \nabla J\left(\phi \right)=E_{s∼S,a∼A}\left[\nabla_{\phi }\log\;\pi_{\phi }\left(a|s\right)A^{\pi_{\phi }}\left(s,a\right)\right]. \end{array}$$

Subtracting *Q*^*π*_*ϕ*_^ by *V*^*π*_*ϕ*_^ gives the advantage function *A*^*π*_*ϕ*_^ used in equation (4):

(5) $$\begin{array}{c} A^{\pi_{\phi }}\left(s,a\right)=Q^{\pi_{\phi }}\left(s,a\right)-V^{\pi_{\phi }}\left(s\right), \end{array}$$

where *A*^*π*_*ϕ*_^(*s*, *a*) reflects the expected additional reward that the agent will receive after taking action *a* at state *s*.

To evaluate the generalization capability of demonstrations [7], we should firstly define different MDPs within the RLfD paradigm, where the source MDP ℳ_*s*_: 〈*𝒮*_*s*_, *𝒜*_*s*_, ℛ_*s*_, *𝒫*_*s*_, *γ*〉 is used to collect the expert demonstrations and ℳ_*t*_: 〈*𝒮*_*t*_, *𝒜*_*t*_, ℛ_*t*_, *𝒫*_*t*_, *γ*〉 is the target MDP that needs to be solved. In RLfD, an RL agent interacts with the environment following the target MDP ℳ_*t*_ and is also provided with expert demonstrations generated by the expert policy *π*_*E*_ from source MDP ℳ_*s*_. In RL, the generalization settings can be various, where ℳ_*s*_ and ℳ_*t*_ can differ by state space *𝒮*, action space *𝒜*, reward function ℛ, or system dynamics *𝒫*.

As a generalization of the standard MDP, the partial observable Markov decision process (POMDP) [33] extends MDP to the partial observable environment settings. In POMDP, the agent only receives an observation *o*_*t*_ with distribution *p*(*o*_*t*_*|s*_*t*_) at each time step *t*. Similar to the standard MDP, the aim of the POMDP is to maximize the expected total reward that the RL agent receives. Moreover, the other core issue in POMDP is to improve the robustness of the trained policy to the stochastic disturbance of the environment.

### 3.2. Bayesian Networks

Bayesian networks [9] belong to probabilistic graphical models (PGMs) that can be defined as 〈*𝒢*, *𝒪*〉 where *𝒢*=(*𝒱*, *ℰ*) is the directed acyclic graph, with *𝒱* is the set of nodes (variables) and edges *ℰ*, and *𝒪* is the probability function. Depending on whether the variables are discrete or continuous, Bayesian networks can be classified into discrete Bayesian networks and Gaussian Bayesian networks. In addition to Gaussian distribution, alternative techniques such as modified exponential distribution and Rayleigh distribution can also be used to deal with continuous attributes [34]. Since only discrete Bayesian networks are employed in this paper, we use Bayesian networks to represent discrete Bayesian networks in the following paper for convenience. To utilize a Bayesian network, both the structure *𝒢* and probability function *𝒪* of the Bayesian network should be obtained, where *𝒪* is quantified by a conditional probability table (CPT) that can be parameterized by *θ*. Depending on the characteristics of the task to be solved, the topology *𝒢* can either be defined based on the causality of nodes or learned from data. For most RL tasks, since the state inputs and action outputs are known, the causal relationship between states and actions can be directly described by a Bayesian network structure (see also Figure 2). Thus, we focus on estimating the optimal parameter *θ*^*∗*^ of the probability function and the probabilistic inference of Bayesian networks.

#### 3.2.1. Parameter Estimation

The parameter estimation process of Bayesian networks aims to learn the probability function *𝒪* of all the nodes, where each node in Bayesian networks denotes a variable [35]. Providing the structure *𝒢* of a Bayesian network, the conditional independence of all the nodes can be learned from data. Given a dataset *𝒟* consists of fully observed samples of a Bayesian network, the maximum likelihood estimation (MLE) method is usually used to accomplish the parameter estimation process. Suppose a Bayesian network has *n* nodes **X**={*X*_1_, *X*_2_,…, *X*_*n*_} and its probability function *𝒪* is parameterized by *θ*. For the node *X*_*i*_ in **X**, we assume that it has *r*_*i*_ candidate values and its parent nodes parent(*X*_*i*_) have *q*_*i*_ candidate combinations. Each parameter *θ*_*ij*_^*k*^ that represents the conditional probability between node *X*_*i*_ and its parent nodes parent(*X*_*i*_) when *X*_*i*_=*k* and parent(*X*_*i*_)=*j* can be written as

(6) $$\begin{array}{c} \theta_{ij}^{k}=P\left(X_{i}=k|\text{parent}\left(X_{i}\right)=j\right), \end{array}$$

where *i*=1,2,…, *n*; *j*=1,2,…, *q*_*i*_; *k*=1,2,…, *r*_*i*_.

According to the property of probability, the accumulated sum of *θ*_*ij*_^*k*^ over candidate values of *X*_*i*_ satisfies

(7) $$\begin{array}{c} \sum_{k=1}^{r_{i}}\theta_{ij}^{k}=\sum_{k=1}^{r_{i}}P\left(X_{i}=k|\text{parent}\left(X_{i}\right)=j\right)=1. \end{array}$$

The MLE method aims at learning the optimal parameter *θ*^*∗*^ by maximizing the likelihood between the parameter *θ* and the dataset *𝒟*, which can be written as

(8) $$\begin{array}{c} \theta^{*}=\text{arg}\underset{\theta }{\max}L\left(\theta |D^{E}\right)=\text{arg}\underset{\theta_{ij}^{k}}{\max}\sum_{i=1}^{n}\sum_{j=1}^{q_{i}}\sum_{k=1}^{r_{i}}m_{ij}^{k}\log\;\theta_{ij}^{k}, \end{array}$$

where *L*(*θ|𝒟*) is the likelihood function of *θ* and *m*_*ij*_^*k*^ is the number of samples that satisfies parent(*X*_*i*_) when *X*_*i*_=*k* and parent(*X*_*i*_)=*j* in the dataset *𝒟*.

By using the Lagrange multiplier method, the (near) optimal *θ*^*∗*^ can be obtained as follows:

(9) $$\begin{array}{c} \theta_{ij}^{k*}=\left\{\begin{array}{cc} \frac{1}{r_{i}}, & \text{if }\sum_{k=1}^{r_{i}}m_{ij}^{k}=0,\\ \frac{m_{ij}^{k}}{\sum_{k=1}^{r_{i}}m_{ij}^{k}}, & \text{if }\sum_{k=1}^{r_{i}}m_{ij}^{k}>0. \end{array}\right. \end{array}$$

Recently, some advanced Bayesian network parameter estimation methods are also proposed for limited data [36] or uncertain data [37]. As we have enough deterministic data and the MLE method has high estimation accuracy and wide application, we choose MLE as the method for parameter estimation in this paper.

#### 3.2.2. Probabilistic Inference

The probabilistic inference of Bayesian networks is to estimate the posterior probability on target variables by giving the learned CPTs and observed variables (also called evidence variables), which can be divided into approximate inference and exact inference. Exact inference methods aim to precisely calculate the probability distribution of variables and are suitable for Bayesian networks with simple structures. Approximate inference methods improve the computational efficiency at precision, which is suitable for Bayesian networks with complex structures.

Given the structure of a Bayesian network example shown in Figure 2, its joint probability distribution can be written as

(10) $$\begin{array}{c} P\left(x,\dot{x},\psi ,\dot{\psi },a\right)=P\left(x\right)\cdot P\left(\dot{x}\right)\cdot P\left(\psi \right)\cdot P\left(\dot{\psi }\right)\cdot P\left(a|x,\dot{x},\psi ,\dot{\psi }\right), \end{array}$$

where *P*(·) denotes the probability distribution function.

Since the structures of Bayesian networks used in this paper are relatively uncomplicated, we can choose exact inference methods without having to sacrifice the accuracy for computational efficiency. As one of the representative exact inference methods, variable elimination (VE) can decompose the joint probability distribution, and the Bayesian network represents into a series of conditional probability products and accomplishes the inference process by integration. Therefore, giving the goal of obtaining the marginal probability *P*(*a*), the VE method eliminates variables *x*, $\dot{x}$, *ψ*, and $\dot{\psi }$ in equation (10) as follows:

(11) $$\begin{array}{c} P\left(a\right)=\sum_{\dot{\psi }}\sum_{\psi }\sum_{\dot{x}}\sum_{x}P\left(x,\dot{x},\psi ,\dot{\psi },a\right)\\ =\sum_{\dot{\psi }}\sum_{\psi }\sum_{\dot{x}}\sum_{x}P\left(x\right)\cdot P\left(\dot{x}\right)\cdot P\left(\psi \right)\cdot P\left(\dot{\psi }\right)\cdot P\left(a|x,\dot{x},\psi ,\dot{\psi }\right). \end{array}$$

## 4. Methodology

In this section, firstly a novel state abstraction algorithm called node influence with Wasserstein distance (NIW) is proposed. Given the learned abstract states, the probabilistic knowledge extraction method with Bayesian networks is introduced in Section 4.1. Then, our RLBNK method that incorporates such probabilistic knowledge into RL is presented in Section 4.2. More specificity, two variant extensions of the RLBNK method, RLBNK-concat and RLBNK-switch, are designed for different knowledge integration approaches. Finally, we analyse and discuss the advantages of our RLBNK method in Section 4.3.

### 4.1. Extracting Probabilistic Knowledge by Bayesian Networks

In previous RLfD methods, demonstrations are certain instances of human knowledge for a specific task. In order to improve their generalization capability and robustness, higher-level knowledge should be extracted from demonstrations first. Since the number of demonstrations is usually insufficient to cover the entire statespace of a task, and human knowledge is naturally coarse and probabilistic, providing uncertainty in instructions is essential to utilize demonstrations well. As Bayesian networks have the advantages of extracting and representing probabilistic knowledge and are interpretable, we choose this pattern for the knowledge representation.

#### 4.1.1. State Abstraction via NIW Algorithm

Since Bayesian networks only take discrete variables as input and output, the state abstraction should be obtained before the probabilistic knowledge extraction process, which can be done by discretization. In addition to being used to build Bayesian networks, discrete states have the advantage of being easier to understand and closer to conceptual and semantic representations than continuous states. Furthermore, the discrete state can contribute to the robustness of the learned policy compared to the original continuous state.

For convenience, we take the CartPole task as an example here and other tasks used in this paper are similar. The state vector of the CartPole task is $\left[x,\dot{x},\psi ,\dot{\psi }\right]$, which represents the position and the velocity of the cart, and the angle and the angular velocity of the pole, respectively. In order to acquire the state abstraction, each state element is semantically divided into Negative, Small, and Positive. The discretization process follows equation (12), where *δ*_*i*_ denotes the parameter of discretization for each state element *s*_*i*_ in state vector. For example, *δ*_*x*_, $\delta_{\dot{x}}$, *δ*_*ψ*_, and $\delta_{\dot{\psi }}$ indicates the discretization parameter for each state element in $\left[x,\dot{x},\psi ,\dot{\psi }\right]$ for the CartPole task:

(12) $$\begin{array}{c} S_{i}=\left\{\begin{array}{cc} \text{Small}, & \text{if }\left|s_{i}\right|<\delta_{i},\\ \text{Positive}, & \text{if }s_{i}\geq \delta_{i},\\ \text{Negative}, & \text{if }s_{i}\leq -\delta_{i}. \end{array}\right. \end{array}$$

Different *δ*_*i*_ for discretization would result in different representations of states, which can significantly affect the learning and inference process of Bayesian networks. Previous work has shown that abstract concepts can be learned from similarity-based approach [38], where the *δ*_*i*_ is determined by the similarity. Oller et al. [39] proposes a concept learning method via clustering to implicitly find. However, this unsupervised approach does not consider the causal relationships between variables.

In Bayesian networks, the optimal state abstraction parameter *δ*_*i*_ should enable the most efficient prediction and inference capacity, which can be measured by the node influence [40, 41]. The node influence value stands for the discrepancy of conditional and marginal probabilities of the target probability distribution, which indicates the inference ability between variables. Based on this idea, we propose a novel state abstraction algorithm called node influence with Wasserstein distance (NIW) to find the optimal *δ*_*i*_. NIW quantifies the relationship between two causal variables by describing the variability of the target probability distribution. A larger NIW value indicates a stronger inference capability between variables. We calculate the NIW value as follows:

(13) $$\begin{array}{c} \text{NIW}=\frac{1}{u}\cdot \sum_{i=1}^{u}\eta \cdot D_{W}\left(P\left(Y\right)|,|P|\left(Y|X=x_{i}\right)\right), \end{array}$$

where *X* is the parent node of *Y* (See Figure 3), *u* is the number of discretized states, *D*_*𝒲*_(·, ·) is the Wasserstein distance metric, and *η* is the ratio of the samples that satisfy *X*=*x*_*i*_.

The Wasserstein distance can be calculated by

(14) $$\begin{array}{c} D_{W}\left(p,q\right)=\underset{\gamma \in \Pi \left[p,q\right]}{\inf}\iint \gamma \left(x,y\right)\text{d}\left(x,y\right)\text{d}x\text{d}y, \end{array}$$

where *γ*(*x*, *y*) satisfies

(15) $$\begin{array}{c} \int \gamma \left(x,y\right)\text{d}y=p\left(x\right),\\ \int \gamma \left(x,y\right)\text{d}x=q\left(y\right), \end{array}$$

and d(*x*, *y*) satisfies

(16) $$\begin{array}{c} \text{d}\left(x,y\right)={\left\|x-y\right\|}_{2}=\sqrt{\sum_{i=1}^{n}{\left(x_{i}-y_{i}\right)}^{2}}. \end{array}$$

In contrast to the Kullback–Leibler divergence metric and the Jensen–Shannon divergence metric, the Wasserstein distance [42] metric can measure not only the distance between two overlapping distributions, but also the distance between two nonoverlapping distributions, which provides more useful information for evaluating the relationships of variables in Bayesian networks. By calculating the NIW values corresponding to a series of different *δ*_*i*_, we can determine that the one corresponding to the maximum NIW value is the optimal *δ*_*i*_.

#### 4.1.2. Knowledge Extraction via Bayesian Networks

After determining *δ*_*i*_ by calculating the NIW value for discretization, the probabilistic knowledge can be extracted from data via Bayesian networks, where the knowledge extraction process is also referred to as the parameter estimating of Bayesian networks. The workflow of probabilistic knowledge extraction is shown in Figure 4. Given the discretization parameters and the original dataset *𝒟*^*E*^ which contains continuous state variables, the original state should be firstly abstracted to *𝒟*_abstract_^*E*^ following equation (12). As the structure of the Bayesian network is known, the parameter of Bayesian network can be estimated according to equation (9) with abstract dataset *𝒟*_abstract_^*E*^.

The pseudocode of the knowledge extraction process for this section is shown in Algorithm 1.

**Remark 1 .**

According to equation (11) and equation (13), the computational complexity of Algorithm 1 can be estimated as *𝒪*(*n*^2^2^*k*^), where *n* is the number of nodes in the Bayesian network and *k* is the maximum number of parent nodes.

### 4.2. Incorporating Probabilistic Knowledge into Reinforcement Learning

As the Bayesian network represents the knowledge extracted from demonstrations, we use the knowledge module *𝕂*_*θ*^*∗*^_ to refer to it for convenience, where *θ*^*∗*^ is learned following Algorithm 1. The knowledge module *𝕂*_*θ*^*∗*^_ outputs the decision confidence vector **p** that indicates the uncertainty estimation of the decisions, therefore to determine the extent to which the decision should be trusted. Formally, the output vector **p** of the probabilistic knowledge module *𝕂*_*θ*^*∗*^_ is based on the current state *s* following equation (11) and it can be written as

(17) $$\begin{array}{c} p=K_{\theta^{*}}\left(s\right)=\left[p_{a_{1}},p_{a_{2}},\ldots ,p_{a_{\left|A\right|}}\right], \end{array}$$

where *p*_*a*_*i*__ is the decision confidence over action *a*_*i*_ and the sum of all the *p*_*a*_*i*__ satisfies: ∑_*i*=1_^|*𝒜*|^*p*_*a*_*i*__=1.

**Definition 1 .**

In RL paradigm, the knowledge extracted by Bayesian networks can be formally defined by a tuple 〈*S*_*𝕂*_, *𝕂*_*θ*_〉, where *𝒮*_*𝕂*_⊆*𝒮* is the state space that the knowledge module *𝕂*_*θ*_ works and *𝕂*_*θ*_ is a mapping from *𝒮*_*𝕂*_ to action space *𝒜* with high decision confidence.

Even though the knowledge module *𝕂*_*θ*^*∗*^_ plays the role of probabilistic knowledge extraction and representation, the knowledge extracted from demonstrations is still coarse and needs to be further extended and refined. Therefore, a knowledge refine module *𝔽*_*ϕ*_ should be introduced, which should at least take the decision confidence vector **p** as the input and outputs the refined decision confidence vector **p**′. As a flexible universal approximator, a neural network can be combined with other patterns, including Bayesian networks, to form hybrid policies *π*_hybrid_. Thus, we use a neural network-based refine module *𝔽*_*ϕ*_ here to undertake the role of knowledge refinement and propose two alternative RLBNK methods: RLBNK-concat and RLBNK-switch to approximate the refine module.

#### 4.2.1. RLBNK-Concat

With the decision confidence vector **p** provided by the knowledge module *𝕂*_*θ*^*∗*^_, the first idea of incorporating knowledge into the RL process is to directly concatenate the vector **p** to the current state *s* as the input of the refine module *𝔽*_*ϕ*_. This idea indiscriminately considers both the current state and the decision confidence. By concatenating these two vectors as the input of the refine module, the output refined action preference vector **p**′ can be obtained from the output of the refine module following

(18) $$\begin{array}{c} p^{\prime }=F_{\phi }\left(p,s\right)=\left[p_{a_{1}}^{\prime },p_{a_{2}}^{\prime },\ldots ,p_{a_{\left|A\right|}}^{\prime }\right]. \end{array}$$

For this RLBNK-concat method, we define its whole policy can be represented as *π*_hybrid_^*c*^=*𝕂*_*θ*^*∗*^_ ⊗ *𝔽*_*ϕ*_, where the policy *π*_hybrid_^*c*^ will be optimized within the RL paradigm. Since the parameter *θ*^*∗*^ is learned via Algorithm 1, only the parameter *ϕ* of the refine module will be optimized during the policy optimization process. Although the RLBNK-concat method is straightforward and feasible, it does not fully leverage the decision confidence **p** provided by the knowledge module, which results in the refine module *𝔽*_*ϕ*_ having to function in the domain with size |*𝒮*|+|*𝒜*|, while the original size of the state space is |*𝒮*|. However, when the RL agent encounters states in which it has a high decision confidence based on prior knowledge, it can rely solely on the prior knowledge to complete the decision-making process without further learning.

#### 4.2.2. RLBNK-Switch

As shown in Figure 5, to better utilize the decision confidence provided by the knowledge module *𝕂*_*θ*^*∗*^_, we propose RLBNK-switch by comparing the action confidence *p*_*a*_*i*__ with the threshold ∧ to determine the source of decisions following equation (19). More specifically, we can choose whether the action should be taken from the knowledge module or from the refine module according to decision confidence values *p*_*a*_*i*__. If the decision confidence is high, the decision will be made based on the prior knowledge module *𝕂*_*θ*^*∗*^_. Otherwise, the agent can switch to the refine module *𝔽*_*ϕ*_ to make the decision, where the refine module will be further optimized by RL. Therefore, comparing to RLBNK-concat, the RL agent only learns the policy in states that are uncovered by the knowledge module. The switching process can be expressed as

(19) $$\begin{array}{c} p^{\prime }=\left\{\begin{array}{cc} p, & \text{if }\max\left(p\right)>\wedge ,\\ F_{\phi }\left(s\right), & \text{else,} \end{array}\right. \end{array}$$

where max(·) is used to return the maximum element of the input vector.

For RLBNK-switch, we define its whole hybrid policy can be represented as *π*_hybrid_^*s*^=*𝕂*_*θ*^*∗*^_⊙*𝔽*_*ϕ*_. After obtaining the refined action preference vector, the action *a*_*i*_ should be taken if the corresponding decision confidence *p*_*a*_*i*__′ is the maximum element in the output vector **p**′. Then, the whole policy *π*_hybrid_^*s*^ will be optimized. Since the parameter *θ*^*∗*^ is fixed, only the neural network refine module *𝔽*_*ϕ*_ will be optimized following the policy optimization procedure in RL based on equation (3).

**Remark 2 .**

Assuming that the learned knowledge module *𝕂*_*θ*^*∗*^_ is the optimal policy in state space (domain) *𝒮*_*𝕂*_, because of the switch mechanism of the RLBNK-switch method, the hybrid policy *π*_hybrid_^*s*^ is optimal in state space *𝒮*_*𝕂*_ but is nonoptimal in state space *𝒮* − *𝒮*_*𝕂*_. From a holistic point of view, the hybrid policy *π*_hybrid_^*s*^ has an optimal initialization for partial state space, which makes this RLBNK-switch method have the same feasibility as the normal neural network-based RL algorithms.

As the proposed RLBNK method can be regarded as a general policy framework where it can be represented by *π*_hybrid_^*c*^ = *𝕂*_*θ*^*∗*^_ ⊗ *𝔽*_*ϕ*_ (for RLBNK-concat) or *π*_hybrid_^*s*^ = *𝕂*_*θ*^*∗*^_⊙*𝔽*_*ϕ*_ (for RLBNK-switch), the RLBNK method is able to combine with any policy-based RL algorithm to optimize the parameter *ϕ* of the refine module *𝔽*_*ϕ*_. As the proximal policy optimization (PPO) [43] algorithm is considered as a baseline RL algorithm, we apply it as the base algorithm in this paper to demonstrate the effectiveness of RLBNK.

The PPO algorithm has two variant versions and the most commonly used version is the one with clipped surrogate objective, which forms the policy gradient using the advantage function *A*^*π*_*ϕ*_^ as introduced in equation (5) and minimizes the clipped-ratio loss *L*^PPO^(*ϕ*) over samples collected by *π*_*ϕ*_old__. The clipped-ratio loss can be written as

(20) $$\begin{array}{c} L_{t}^{\text{PPO}}\left(\phi \right)=E_{\left(s,a\right)∼\pi_{\phi_{\text{old}}}}\left[\min\left(\rho \left(\phi \right)A_{t}^{\pi_{\phi }},\text{clip}\left(\rho \left(\phi \right),1-\varepsilon ,1+\varepsilon \right)A_{t}^{\pi_{\phi }}\right)\right], \end{array}$$

where the clipping coefficient *ϵ* aims to prevent large updates. The probability ratio *ρ*_*t*_(*ϕ*) used in equation (20) is introduced to measure the changed probability of the chosen action *a* in state *s* under the updated policy *π*_*ϕ*_ and the old policy *π*_*ϕ*_old__, which can be written as

(21) $$\begin{array}{c} \rho \left(\phi \right)=\frac{\pi_{\phi }\left(a|s\right)}{\pi_{\phi_{\text{old}}}\left(a|s\right)}. \end{array}$$

For the policy network in PPO, the overall loss function at time step *t* is defined by the combination of the surrogate loss *L*^PPO^(*ϕ*), the value loss *L*^VF^(*ϕ*), and the entropy *K*. The weights of these items are adjusted by coefficients *c*_1_ and *c*_2_:

(22) $$\begin{array}{c} L_{t}\left(\phi \right)={\hat{E}}_{t}\left[L_{t}^{\text{PPO}}\left(\phi \right)+c_{1}L_{t}^{VF}\left(\phi \right)-c_{2}K\left[\pi_{\phi }\right]\left(s\right)\right]. \end{array}$$

The weights of neural networks can be updated as follows:

(23) $$\begin{array}{c} \phi ⟵\phi +\alpha \frac{\partial L_{t}\left(\phi \right)}{\partial \phi }. \end{array}$$

The pseudocode of RLBNK is shown in Algorithm 2.

### 4.3. Performance Analysis and Discussion

The RLBNK method can be regarded as the neurosymbolic AI where the Bayesian network is the symbolic representation of knowledge while the refine module is represented by the neural network. Symbolism is expected to provide extra knowledge constrains for the learning process to help improve the learning efficiency, which can also prevent the well-known catastrophic forgetting of neural networks and the difficulty of extrapolation nondistributed data to improve the robustness of the algorithm [26, 44].

#### 4.3.1. Efficiency Analysis

Formally, for the MDP defined by 〈*𝒮*, *𝒜*, ℛ, *𝒫*, *γ*〉, the size of its policy space is |*𝒜*|^|*𝒮*|^. Assuming that the knowledge module provides high decision confidence values in state set *𝒮*_*𝕂*_, where *𝒮*_*𝕂*_⊆*𝒮*, the policy space of the refine module *𝔽* for RLBNK-switch is reduced from |*𝒜*|^|*𝒮*|^ to |*𝒜*|^|*𝒮* − *𝒮*_*𝕂*_|^. Therefore, the uncertainty-based state space partitioning can make RLBNK-switch theoretically enjoy better data efficiency performance. Additionally, the knowledge module can cover the policy space |*𝒜*|^|*𝒮*_*𝕂*_|^, which is fixed to prevent the catastrophic forgetting as well as reducing the overall policy space that needs to be learn. And the knowledge represented by Bayesian networks provides better generalization and robustness over the neural network-based method because of the state abstraction and the probabilistic property of Bayesian networks. For RLBNK-switch, the RL algorithm is employed to learn a policy for the state space *𝒮* − *𝒮*_*𝕂*_. Therefore, the gradient estimator also turns from equation (4) into

(24) $$\begin{array}{c} \nabla J\left(\phi \right)=E_{s∼\left(S-S_{K}\right),a∼A}\left[\nabla_{\phi }\log\;\pi_{\phi }\left(a|s\right)A^{\pi_{\phi }}\left(s,a\right)\right], \end{array}$$

which also avoids an integral over the full state space to make the learning more efficient. Moreover, for RLBNK-concat, because of the concatenation operation, the policy space is increased from |*𝒜*|^|*𝒮*|^ to |*𝒜*|^|*𝒮*|+|*𝒜*|^. Therefore, we expect that RLBNK-switch method demonstrates a better data efficiency performance than RLBNK-concat.

#### 4.3.2. Robustness Analysis

Conditional independence used in Bayesian networks is the basic and robust form of knowledge. The Bayesian network classifier is robust, and we can learn the parameters of conditional distribution even with relatively few training examples [35]. Also, the variance that Bayesian networks provide makes them act robust. Besides, in our paper, the knowledge are constrained by the threshold ∧, which also improves the robustness. The state abstraction (discretization) NIW method also plays an important role to improve the robustness. Discrete values are about intervals of numbers which are more concise to specify, easier to use, and comprehend as they are closer to a concept-level representation than continuous ones [45, 46]. From the perspective of machine learning, state abstraction reduces the risk of overfitting by minimizing structural risk and eliminates noisy samples by simplifying the data, both of which enhance the robustness and generalization capability.

## 5. Experiments

In this section, we conduct experiments to evaluate our RLBNK method. More specifically, for the experiments below, we aim to evaluate our proposed RLBNK method to confirm the following:

- Our RLBNK method contributes to the data efficiency of RL under the normal reward setting and even sparse reward settings.
- The knowledge extracted from demonstrations through Bayesian networks can be generalized to similar tasks, providing instructive guidance for the RLBNK method to obtain effective hybrid policies.
- With the help of the knowledge learned by Bayesian networks, the hybrid policy *π*_hybrid_ learned by the RLBNK method can robustly handle noisy observations from the environment.

All the experiments in this paper are conducted in the Ubuntu 16.04 system with PyTorch 1.7. Our algorithms are based on the open-source PPO-PyTorch [47] implementation and the probabilistic graphical model toolkit pgmpy [48]. We test our algorithms on the OpenAI Gym [49] environment and the PLE [50] environment. Below we briefly describe the tasks used in our experiments (also see Figure 6).

 
*CartPole*. In the CartPole system, a cart moves along a friction-less track and the pole is attached by an unactuated joint to the cart. The goal of this task is to balance the pole vertically upward as long as possible.
 
*Catcher*. In the Catcher task, the paddle has to catch the falling fruit with three different actions (moving left, moving right, and doing nothing), the RL agent has access to the position and speed of both the player and the fruit.
 
*FlappyBird*. FlappyBird is a side-scrolling game where the bird takes actions (flapping or doing nothing) to fly through gaps between pairs of pipes. The agent receives the reward once the bird passes through a pipe and the episode ends when the bird hits pipes or gets out of the screen.

### 5.1. Simulation Settings

To ensure the fairness of our experiments, we keep all the hyperparameters the same as the original implementation as recommended in the corresponding literature. For CartPole and Catcher task, 2000 state-action pairs (*s*, *a*) are collected by an expert policy *π*_*E*_to form the original expert demonstration dataset *𝒟*^*E*^, and for FlappyBird task, 150 state-action pairs are collected via the same way. Specially, the update interval of networks *T*_update_ is set to 2000, and the clipping parameter *ϵ* for policy optimization is set to 0.2. All the neural networks used in this paper have 2 hidden layers, each containing 64 neurons. The optimal discretization parameters *δ*_*i*_ for state abstraction during the knowledge extraction process are are shown in the tables in Appendix, where the parameter corresponding to the maximum NIW value is the optimal parameter for subsequent experiments. For RLBNK-switch, the knowledge module threshold parameter ∧ is set to 0.8 as default. For each algorithm and each task, we train 5 policies with different seeds and the shaded region for each curve in the following results denotes the standard deviation of the average evaluation.

### 5.2. Data Efficiency of the RLBNK Method

To evaluate the validity of the proposed RLBNK method, we first conduct experiments on three tasks mentioned above under the normal reward setting. To further demonstrate the effectiveness of the proposed RLBNK method, we also set up CartPole tasks with variant sparse reward settings. The performance under different reward settings is shown in Figures 7 and 8, respectively.

#### 5.2.1. Performance Comparison under the Normal Reward Setting

Curves in Figure 7 illustrate the mean and variance of the cumulative reward in each episode for the training process of RLBNK-switch, RLBNK-concat, baseline PPO [43], and DQfD [16] in these tasks. The Expert curve denotes the performance of the expert policy *π*_*E*_ used to collect demonstrations, and the Imitation curve is the performance of the policy trained using demonstrations via behavior cloning [11].

From Figure 7, we can observe that both proposed RLBNK-switch and RLBNK-concat outperform other baseline methods in most cases and RLBNK-switch demonstrates a jump-start for all three tasks at the beginning of each training process. Both proposed algorithms obtain higher rewards within fewer training episodes. Especially, the performance of RLBNK-switch in all three tasks learns a good (even near optimal) policy within 200 episodes. Compared to the baseline algorithm PPO that explores the environment from scratch, our method is superior by leveraging the knowledge extracted from demonstrations. In contrast, although the DQfD method utilizes the same demonstration data as RLBNK-switch and RLBNK-concat, it performs mediocrely in all cases except for the CartPole task where it outperforms than RLBNK-concat. We assume this is because the reward setting in Catcher and FlappyBird is relatively sparser than the CartPole task and this will be further analysed in the next experiment. This result confirms that the proposed RLBNK method can effectively utilize the knowledge and achieve superior performance.

#### 5.2.2. Performance Comparison under Sparse Reward Settings

We further demonstrate the superiority of RLBNK-switch and RLBNK-concat under sparse reward conditions. To facilitate experimental validation, we propose a sparse reward setup: multistep cumulative rewards are given at sparse time steps. We choose the CartPole task to simulate this setup and provide *T*-step cumulative rewards at every *T* time step (the rewards are only provided at *T*, 2*T*, 3*T*,…).  Figure 8 shows the experimental results under different sparse settings.

From Figure 8, we can remark that our RLBNK-switch converges within around 200 episodes and demonstrates smaller variance a consistent performance for all three sparse settings ranging from 25 to 100. The baseline PPO is hard to learn an effective policy under sparse reward settings since the PPO agent has less chance to obtain reward signals in the early pure exploration phase of learning. For DQfD, even if it achieves a good preference under normal reward setting in CartPole task, it acts the worse learning process in all sparse settings. We believe that one possible reason is that the priority sampling mechanism used by the DQfD algorithm hinders the Q-network updates under sparse reward conditions. This priority sampling mechanism gives more priority to demonstrations during the Q-network update process. However, due to sparse reward settings, the DQfD agent has difficulty obtaining positive samples from the environment itself, so the Q-network in DQfD may still be optimized with pure demonstrations for most of the time, even though the agent is interacting with the environment. Since demonstrations only cover part of the state space, it cannot optimize the Q-network well enough to obtain a well-performed policy. Moreover, from the learning curves shown in Figure 8, for DQfD and baseline PPO, the task becomes harder as the sparse factor *T* increases, while both RLBNK-switch and RLBNK-concat are less influenced.

### 5.3. Evaluation of the Generalization Capability

In this section, we perform experiments to examine the generalization capability of the RLBNK method. Here, we focus on the generalization settings that ℳ_*s*_ and ℳ_*t*_ share the same state space *𝒮*, action space *𝒜*, and reward function ℛ but differ by the system dynamics: *𝒫*_*s*_ ≠ *𝒫*_*t*_. Specifically, we adopt the CartPole task here and change the length of the pole and the mass of the cart for the generalization settings as shown in Table 1. Note that given the demonstrations collected in the source MDP ℳ_*s*_, our aim is to solve the target MDP ℳ_*t*_.

In this experiment, we carry out several baselines, including PPO [43], PPO-finetune, DQfD [16], and Imitation (via supervised behavior cloning [11]). The PPO-finetune curve denotes the performance of the RL policy pretrained by PPO in the source MDP ℳ_*s*_ and then fine-tuned in the target MDP ℳ_*t*_. The PPO curve illustrates the performance of the baseline PPO directly trained in the target MDP ℳ_*t*_. DQfD utilizes the demonstrations collected in the source MDP and explores in the target MDP. In the Imitation curve, the corresponding policy is trained with the expert demonstrations collected from the source MDP ℳ_*s*_ via supervised behavior cloning. The curve shows its performance in the target MDP ℳ_*t*_.

From Figure 9, it can be observed that in both generalization settings, directly imitating the demonstrations collected from the source MDP ℳ_*s*_ cannot achieve a good performance in the target MDP (as shown in the Imitation curve). In contrast, RLBNK-switch achieves the best performance and with the help of the knowledge learned from source MDP, and both RLBNK-switch and RLBNK-concat outperform the baseline PPO algorithm. Since the policy in the PPO-finetune method is initialized as a well-trained policy in the source MDP and fine-tunes in the target MDP, it is a powerful method that achieves comparable performance to RLBNK-concat in the pole length generalization settings and even surpasses the RLBNK-concat in the cart mass generalization settings. In contrast, the DQfD method demonstrates the worse performance in both settings. One possible reason is that after the pretraining process, the demonstrations collected from the source MDP, although not suitable for the target MDP, are still used indiscriminately to update the Q-network, which hinders its optimization process in the target MDP. The empirical results in both pole length generalization and cart mass generalization show the strong evidence that the proposed RLBNK-switch achieves superior performance in generalization settings and the RLBNK-concat also demonstrates a comparable result to the PPO-finetune method. RLBNK-switch and RLBNK-concat can not only improve the data efficiency but also can generalize to tasks with different system dynamics.

### 5.4. Robustness against Stochastic Disturbances

To make the learned policy achieve robustness against stochastic observation disturbances is one of the goals of POMDP. We extensively evaluate the robustness of the RLBNK method in the CartPole task by injecting stochastic disturbance *ζ* to the state *s*, and the observation *o*_*t*_ satisfies

(25) $$\begin{array}{c} o_{t}=s_{t}+\zeta , \end{array}$$

where *ζ* is sampled uniformly from the set *U*: *U*(0, Φ)={*ζ* : ‖*ζ*‖_*∞*_ ≤ Φ} and the disturbance strength Φ denotes the upper bound of the stochastic disturbance. To evaluate the robustness, we firstly conduct baseline PPO, RLBNK-switch, and RLBNK-concat in the CartPole task to obtain their well-performed policies in the environment without noise following the settings introduced in Section 5.1. Then, 500 rollouts are conducted for each trained policy under the environment with a specific noise disturbance strength range from 0.10 to 0.50 to obtain the mean and standard deviation of the cumulative reward.

Figure 10 shows the performance of these policies against stochastic disturbance *ζ*. We can observe that as the disturbance strength Φ increases, the performance of all the learned policies becomes progressively worse. However, our RLBNK method demonstrates better robustness than the learned baseline neural network-based PPO policy for almost all ranges of disturbance strength. Especially, the RLBNK-concat performs significantly better than the RLBNK-switch. We argue that the reason for this phenomenon is due to the fact that the Bayesian network in RLBNK-switch only functions in the state space |*𝒮*_*𝕂*_|, so its robustness works only in this part of the state space. For RLBNK-concat, even though directly concatenating the state *s* and decision confidence vector **p** enlarges the state space for the policy to search, the Bayesian network can provide the robustness for the entire state space.

## 6. Conclusion

In this paper, we develop a novel RLfD method called RLBNK that employs Bayesian networks to extract probabilistic knowledge from expert demonstrations to assist in RL, which provides an alternative perspective of exploiting demonstrations in RLfD. Compared with other RLfD methods, RLBNK utilizes Bayesian networks to extract probabilistic knowledge from demonstrations, which not only enables interpretability of presentation data but also enhances the generalization of the demonstrations. We further extend the RLBNK method to RLBNK-concat and RLBNK-switch and use PPO as the basic policy optimization paradigm. Extensive experiments are conducted on different tasks and the results validate that by utilizing the knowledge module represented by Bayesian networks and the knowledge refine module, both RLBNK-concat and RLBNK-switch outperform other baseline methods in normal reward and sparse reward settings and provides a jump-start at the beginning of the training. More importantly, RLBNK demonstrates a superior performance in generalization settings. Besides, the policy trained by RLBNK is more robust to the environment noise comparing to the policy trained by RL with neural network function approximators. In future work, we will scale our RLBNK to pixel-based decision-making tasks by incorporating feature dimension reduction methods such as variational autoencoders (VAEs).

## Figures and Tables

**Figure 1:** The standard reinforcement learning setup.

**Figure 2:** Structure of the Bayesian network defined for the CartPole task.

**Figure 3:** An example for the NIW value calculation.

**Figure 4:** The probabilistic knowledge extraction process. The parameter estimating of the Bayesian network is based on the *𝒟*_abstract_^*E*^ abstracted from the original dataset *𝒟*^*E*^ via the NIW algorithm.

**Figure 5:** Architecture of the RLBNK-switch method. The knowledge module represented by the Bayesian network is combined with neural network-based refine module according to the decision confidence **p** over the current state.

**Figure 6:** The benchmark tasks used in this paper. The CartPole task is from the OpenAI Gym environment, and the Catcher and FlappyBird tasks are from the PLE environment. (a) CartPole. (b) Catcher. (c) FlappyBird.

**Figure 7:** Comparison of RLBNK-switch and RLBNK-concat to the baseline PPO, DQfD, expert policy, and pure imitation learning under the normal reward setting. Plots show the training performance over the number of episodes. (a) CartPole. (b) Catcher. (c) FlappyBird.

**Figure 8:** Experimental results for CartPole task under different sparse reward settings, where *T* denotes the sparse interval of receiving rewards for the agent. Plots show the training performance over the number of episodes. (a) *T* = 25. (b) *T* = 50. (c) *T* = 100.

**Figure 9:** Comparison of RLBNK-switch and RLBNK-concat to the PPO-finetune, baseline PPO, DQfD, and imitation learning in two generalization settings. Plots show the training performance over the number of episodes. (a) Pole length generalization. (b) Cart mass generalization.

**Figure 10:** The cumulative reward (mean ± standard deviation with 500 rollouts) of RLBNK-switch and RLBNK-concat trained policies versus the trained PPO baseline policy when tested in disturbed CartPole task. Plots show the performance of each policy over the disturbance strength Φ.

**Algorithm 1:** Probabilistic knowledge extraction via Bayesian networks.

**Algorithm 2:** Pseudocode of the RLBNK method.

**Table 1:** The changed system dynamics settings between the source MDP ℳ_*s*_ and the target MDP ℳ_*t*_.

The changed item	Item setting in source MDP	Item setting in target MDP
Pole length (m)	1.0	3.0
Cart mass (kg)	1.0	10.0

**Table 2:** Discretization parameter comparison for the CartPole task.

Position **x**	*δ*_**x**_	0.05	0.10	0.15	0.20	0.25
	NIW	0.064	0.066	**0.068**	0.058	0.043

Velocity $\dot{x}$	$\delta_{\dot{x}}$	0.2	0.4	0.6	0.8	1.0
	NIW	0.028	0.061	0.118	**0.129**	0

Angle *ψ*	*δ*_*ψ*_	0.04	0.05	0.06	0.07	0.08
	NIW	0.054	0.067	**0.095**	0.043	0.065

Angular velocity $\dot{\psi }$	$\delta_{\dot{\psi }}$	0	0.02	0.04	0.06	0.08
	NIW	**0.272**	0.262	0.249	0.172	0.181

**Table 3:** Discretization parameter comparison for the Catcher task.

Distance **x**	*δ*_*x*_	7	9	11	13	15
	NIW	0.079	0.095	**0.117**	0.104	0.103

Height *y*	*δ*_*y*_	34	36	38	40	42
	NIW	0.013	0.019	**0.022**	0.017	0.017

Velocity *v*	*δ*_*v*_	3	4	5	6	7
	NIW	0.101	0.088	**0.114**	0.105	0

**Table 4:** Discretization parameter comparison for the FlappyBird task.

Distance *y*	*δ*_*y*_	0	5	10	15	20
	NIW	**0.192**	0.163	0.090	0.128	0.120

Distance *x*	*δ*_*x*_	20	40	60	80	100
	NIW	0.028	0.048	**0.056**	0.030	0.034

Velocity *v*	*δ*_*v*_	0	2	4	6	8
	NIW	0.206	**0.235**	0.208	0.189	0.020

## Data Availability

The data used to support the findings of this study are included within the article.

## Appendix

Tables 2–4 list the calculated node influence with Wasserstein distance metric (NIW) value with different discretized parameters on datasets collected from three tasks introduced in 5.1. As NIW value reflects the prediction capacity, the threshold parameter corresponding to the maximum NIW value is preferred and will be used in our experiments.
